The article "Study on the Diagnostic Value of Neuroelectrophysiological Examination in Patients with Amyotrophic Lateral Sclerosis" was retracted in 2023. Reasons: signs of a paper mill; compromised peer review; unreliable results or conclusions.

# Study on the Diagnostic Value of Neuroelectrophysiological Examination in Patients with Amyotrophic Lateral Sclerosis

**DOI:** 10.1155/2022/3907751

**Published:** 2022-10-12

**Authors:** Guiyun Ding, Yahua Fan

**Affiliations:** ^1^Department of EMG Laboratory, Nanping First Hospital Affiliated to Fujian Medical University, China; ^2^Department of Neurology, Jian'ou Municipal Hospital of Fujian Province, China

## Abstract

**Objective:**

Amyotrophic lateral sclerosis (ALS) is a progressive neurodegenerative disease with unknown causes involving upper and lower motor neurons. Our study aimed to explore the diagnostic value of neuroelectrophysiological examination in patients with amyotrophic lateral sclerosis.

**Methods:**

A total of 64 patients admitted to our hospital from January 2014 to December 2020 were selected as ALS group. Additionally, 64 normal healthy people in the same period were selected as the control group. Electrophysiological tests were performed on all personnel involved in the study, and the results and parameter changes of different personnel were compared and analyzed.

**Results:**

There was a statistical difference between the EMG data of clinically confirmed ALS and the proposed ALS and possible ALS (*p* < 0.05). The abnormality of confirmed ALS was particularly obvious, and the overall abnormal rate of EMG in ALS was 85%. The CMCT of the upper and lower limbs of clinically diagnosed ALS, suspected ALS, and possible ALS were longer than that of the normal group (*p* < 0.05). There was no significant statistical difference between clinically diagnosed ALS and suspected ALS (*p* > 0.05), and there was a difference between clinically diagnosed ALS and possible ALS (*p* < 0.05). In ALS group, the frequency of F wave decreased, which may be related to the involvement of F wave conduction pathway and the degree of lower motor neuron involvement (*p* < 0.05). In addition, the amplitudes of F and H waves increased, which was related to the involvement of upper motor neurons (*p* < 0.05). In ALS group, SCV was hardly involved, and CMAP decreased significantly, which was positively correlated with the degree of muscular atrophy and muscle strength decline (*p* < 0.05). The sensitivity of electrophysiological detection was 76.56%, the specificity was 78.33%, and the AUC was 0.8578.

**Conclusion:**

Patients with clinically suspected ALS should undergo electrophysiological testing as soon as possible, which is conducive to the early diagnosis and differential diagnosis of ALS. This trial is registered with ChiCTR2100046535.

## 1. Introduction

Amyotrophic lateral sclerosis (ALS) is a progressive neurodegenerative disease with unknown causes involving upper and lower motor neurons. It is the most common type of motor neuron disease [1]. Approximately 70% of patients first present with limb symptoms such as weakness, cramps, and fasciculations, 25% patients with bulbar-onset ALS show dysarthria and dysphagia, and 5% present with initial trunk or respiratory symptoms [2]. As a relentlessly progressive disease, most ALS patients die of respiratory paralysis in 3 to 5 years of diagnosis [3]. In addition, about 50% of patients develop cognitive impairment, 10%-15% of patients meet the diagnostic criteria of frontotemporal dementia (FTD), and ALS patients with FTD have a shorter survival time, which brings a serious burden to patients, their families and society [4, 5].

The article "Study on the Diagnostic Value of Neuroelectrophysiological Examination in Patients with Amyotrophic Lateral Sclerosis" was retracted in 2023. Reasons: signs of a paper mill; compromised peer review; unreliable results or conclusions.

ALS diagnosis is primarily based on clinical assessment and electrophysiological examinations, and repetitive nerve stimulation (RNS) is mainly used to evaluate the function of neuromuscular junction in ALS [6]. ALS image shows the symptoms and signs of upper and lower motor neurons being damaged at the same time, “which is very similar to the clinical image of cervical spondylotic myelopathy (CSM)” or the coexistence of the two diseases. However, the treatment and prognosis of the two diseases are quite different. Early identification of the two diseases is extremely important. Electromyography (EMG) is a time-intensive, operator-dependent diagnostic procedure that requires extensive operator training to become proficient. It is also an important competency for residency training in physical medicine and rehabilitation. EMG training has traditionally been conducted place in a classroom setting, followed by self-study, observation, and finally supervised practical exercises in a clinical setting [7]. Therefore, EMG plays an important role in differentiating ALS from muscle related diseases.

The purpose of this study was to explore the diagnostic value of neuroelectrophysiological detection in patients with amyotrophic lateral sclerosis.

## 2. Materials and Methods

### 2.1. General Clinical Data

A total of 64 patients admitted to our hospital from January 2014 to December 2020 were selected as ALS group. Among the 64 patients, 42 were male and 22 were female; age was 39-72 47.2 ± 8.6 years; the course of disease was 6-72 (48.3 ± 9.5) months; there were 15 cases (22.4%) of bulbar disease, 40 cases (65.5%) of upper limb disease, and 9 cases (12.1%) of lower limb disease. All patients showed slow onset, limb weakness, progressive aggravation, and no obvious limb numbness. Physical examination showed muscle strength decline and muscle atrophy to varying degrees. In this group, there were 52 cases of clinically confirmed ALS, 8 cases of clinically suspected ALS and 4 cases of clinically possible ALS. In addition, 64 normal healthy people in the same period were selected as the control group, including 40 males and 24 females, aged from 40 to 70 years, with an average of 48.95 ± 7.35 years. There was no significant difference in gender and age composition between the two groups. Our study was approved by the Ethics Committee of Nanping First Hospital Affiliated to Fujian Medical University, and all patients signed informed consent.

The article "Study on the Diagnostic Value of Neuroelectrophysiological Examination in Patients with Amyotrophic Lateral Sclerosis" was retracted in 2023. Reasons: signs of a paper mill; compromised peer review; unreliable results or conclusions.

### 2.2. Diagnostic Criteria

According to the diagnostic guidelines of amyotrophic lateral sclerosis in China by the electromyography and clinical neuroelectrophysiology group of the neurology branch of the Chinese Medical Association, the diagnostic grade of ALS is as follows: (1) clinically confirmed ALS: through clinical or electrophysiological examination, it is confirmed that there are 3 or more upper and lower motor neurons involved in 4 regions at the same time; (2) clinically suspected ALS: through clinical or neuroelectrophysiological examination, it is confirmed that there is evidence of simultaneous involvement of upper and lower motor neurons in 2 of the 4 regions; and (3) clinically possible ALS: through clinical or neuroelectrophysiological examination, it is confirmed that there is evidence of simultaneous involvement of upper and lower motor neurons in only one region, or only upper motor neurons in two regions. Imaging and laboratory examinations have been performed to exclude other diseases.

### 2.3. Electrophysiological Detection Method

Using Shanghai Haishen electromyography/evoked potential instrument, electromyography was performed on 3 muscles of upper limbs, bilateral sternocleidomastoid muscles, 2 paraspinal muscles of chest, and 2 muscles of lower limbs in the two groups. Analyze the spontaneous potential, the time limit and amplitude of light force contraction, and the situation and amplitude of strong force contraction; motor evoked potential (MEP) examination of limbs was performed routinely, and the latency, amplitude, and central motor central conduction time (CMCT) of cortical stimulation were analyzed. The frequency and amplitude of F wave response of median nerve, ulnar nerve, and tibial nerve were measured in 38 patients. The amplitude of the H wave recorded in the soleus muscle the motor nerve conduction velocity (MCV), compound muscle action potential (CMAP), distal motor latency (DML), and sensory nerve conduction velocity (SCV), and sensory nerve action potential (SNAP) of median nerve, ulnar nerve, tibial nerve, and peroneal nerve of lower limbs were measured routinely, and the abnormality rate of each index was analyzed.

The article "Study on the Diagnostic Value of Neuroelectrophysiological Examination in Patients with Amyotrophic Lateral Sclerosis" was retracted in 2023. Reasons: signs of a paper mill; compromised peer review; unreliable results or conclusions.

### 2.4. Result Analysis

The abnormal judgment index of electrophysiological examination are as follows: (1) the incubation period was longer than that of the normal group mean +2.5SD. (2) The amplitude decrease was lower than mean-2.5SD in the normal group or the waveform was not drawn out. (3) The increase of wave amplitude was greater than that of normal group mean +2.5SD. (4) The widening of wave duration was greater than that of normal group mean +2.5SD. (5) The difference of bilateral incubation period is greater than mean +2.5SD in the normal group, which is abnormal. (6) The extension of CMCT greater than mean +2.5SD in the normal group is abnormal. (7) Spontaneous potential can be seen in the relaxation state. The light force contraction time limit of EMG > mean +2.5SD is widened, and the amplitude >mean +2.5SD is increased; the recruitment of muscle fibers during vigorous contraction and the measured amplitude >mean+2.5SD were increased.

### 2.5. Statistical Analysis

SPSS 22.0 statistical software was used for processing. Chi-square test was used to compare the counting data. *p* < 0.05 means the difference is statistically significant. ROC curve was used to analyze the sensitivity and specificity of electrophysiological detection of ALS.

## 3. Results

### 3.1. Determination of EMG Value

The EMG measured values are shown in Figure 1. There was a statistical difference between the EMG measured data of clinically confirmed ALS and the proposed ALS and possible ALS (*p* < 0.05). The abnormality of confirmed ALS was particularly obvious, and the overall abnormality rate of EMG in ALS was 85%.

### 3.2. Determination of MEP Value

The values measured by MEP are shown in Figure 2. The CMCT of the upper and lower limbs of clinically confirmed ALS, suspected ALS, and possible ALS were longer than that of the normal group (*p* < 0.05). There was no significant statistical difference between clinically confirmed ALS and suspected ALS (*p* > 0.05), and there was a difference between clinically confirmed ALS and possible ALS (*p* < 0.05). MEP is a sensitivity test for involvement of the pyramidal system. The abnormal rate of CMCT in ALS group was 72.45%, slightly lower than that of EMG.

### 3.3. Comparison of Results of F Wave and H Wave in ALS Group

As shown in Figure 3, the decrease of F wave output rate could be seen in confirmed ALS group (*p* < 0.05), but had no significance in proposed and probably ALS groups, which may be related to the involvement of F wave conduction pathway and the degree of involvement of lower motor neurons. It could also be seen the increased amplitude of F wave and H wave in confirmed ALS groups (*p* < 0.05), but had no significance in proposed and probably ALS groups, which may be related to the involvement of upper motor neurons. In the overall ALS group, the decreased F wave occurrence rate accounted for 33.3%, the increased F wave amplitude accounted for 26.3%, and the increased H wave amplitude accounted for 26.3% (*p* < 0.05).

The article "Study on the Diagnostic Value of Neuroelectrophysiological Examination in Patients with Amyotrophic Lateral Sclerosis" was retracted in 2023. Reasons: signs of a paper mill; compromised peer review; unreliable results or conclusions.

### 3.4. Comparison of Abnormal Rates of Nerve Conduction Values in ALS

As shown in Figure 4, SCV was almost unaffected in ALS group; CMAP and DML were decreased relatively significantly (*p* < 0.05), which was positively correlated with the degree of muscular atrophy and muscle strength decline. The abnormal rate of CMAP accounted for 36.2% of the total ALS group. MCV was slowed down to 4% of the total ALS group, and SNAP was decreased to 3% of the total ALS group (*p* < 0.05).

### 3.5. ROC Curve Analysis of Electrophysiological Detection of ALS

The receiver operating characteristic (ROC) curve of electrophysiological detection was used to evaluate its diagnostic efficacy for ALS. The results showed that the sensitivity of electrophysiological detection was 76.56%, the specificity was 78.33%, and the AUC was 0.8578. It showed that electrophysiological detection of ALS had better diagnostic value, as shown in Figure 5.

## 4. Discussion and Conclusion

In this group of cases, the suspected ALS and possible ALS were confirmed as ALS after half a year to one year of follow-up observation and were incorporated into the ALS database. The abnormal rate of EMG in ALS cases was as high as 85%. EMG remains a basic method to determine the loss of motor units, which include anterior horn cell, motor nerve, neuromuscular junction, and the muscle fibers [8]. In the process of EMG detection, it was found that in patients with early ALS, EMG mostly showed extensive neurogenic damage at three or more sites, so EMG was an important tool to assist in the diagnosis of ALS. However, some patients had atypical symptoms. EMG showed neurogenic damage in only one or two areas, and then neurogenic damage was generalized during follow-up. However, extensive neurogenic damage is also seen in multifocal motor neuron disease, Kennedy disease, cervical spondylosis, etc. [9–13]. EMG is more sensitive to ALS than other examinations, and its specificity should be comprehensively analyzed in close combination with clinical practice after excluding other diseases.

MEP is an important examination for quantitative evaluation of central nervous motor function. ALS cases in this group mainly showed prolonged latency of MEP, decreased or disappeared amplitude of cortical transcranial stimulation, and significantly prolonged CMCT [14]. It is suggested that the motor neuron pool and long motor conduction bundle in the anterior horn of the spinal cord are damaged and the decrease of excitability leads to the disorder of the sum of time and space of indirect wave (I wave) and the amplitude of the wave is significantly reduced or disappeared. MEP shows that the time limit is widened and the conduction time is prolonged. When the fast pyramidal tract fibers are damaged, resulting in the interruption of I-wave conduction, the slow fiber function is retained, and the MEP latency is prolonged. If the slow fiber function is lost, MEP disappears; the decrease in amplitude is mainly due to the activation of the motor neuron pool in the anterior horn cells of the spinal cord and the reduction in the number of neurons [15–17]. The total abnormal rate of MEP in this group was 72.4%, which was significantly higher than that of MCV, F wave and H reflex, with significant statistical difference. In ALS group, MEP in lower limbs was significantly higher than that in upper limbs (*p* < 0.05), and there was also a statistical difference. In nerve conduction measurement, motor nerve abnormality was significantly higher than sensory nerve. Motor nerve abnormality had CMAP decreased significantly, MCV slowed down, DML prolonged, especially CMAP decreased, which was positively correlated with the degree of distal muscular atrophy, and muscle strength decreased, indicating that the loss of motor nerve fibers has been very serious. The main pathological changes of ALS are spinal cord anterior horn cells and axonal degeneration, as well as significant reduction of anterior horn cells. Most of these changes will cause changes in nutritional metabolism and electrophysiology of nerve endings, mainly affecting motor nerves [18]. SCV is basically normal in ALS cases, which is also a characteristic manifestation of ALS. When ALS combined with peripheral nerve entrapment, SCV may be abnormal. Nerve conduction can help ALS differentiate from other peripheral neuropathy [19].

The article "Study on the Diagnostic Value of Neuroelectrophysiological Examination in Patients with Amyotrophic Lateral Sclerosis" was retracted in 2023. Reasons: signs of a paper mill; compromised peer review; unreliable results or conclusions.

F wave mainly reflects the conduction of proximal motor nerve and the function of anterior horn cells, its wave rate reflects the excitability of anterior horn cells, and the central latency to and from the spinal cord reflects the whole pathway [20, 21]. The decrease of F wave output rate is related to the reduction and degeneration of functional cells in the anterior horn of the spinal cord, resulting in the decrease of cell excitability and the reduction of return impulse [22]. The prolongation of F wave latency indirectly indicates the severity of damage to the anterior horn or proximal end of the spinal cord. In this group of cases, it is observed that the frequency of F wave is related to the severity of motor neuron involvement. F wave can be used for the diagnosis of ALS and the evaluation of disease severity [23]. In this group of cases, the abnormal increase of F wave and H wave accounted for 26.3% of the examined nerves, and there were clinical manifestations of upper motor neuron damage. The abnormality of F wave and H wave is not obvious in the early stage of ALS cases. The abnormal increase of F wave and H wave in the middle stage is positively correlated with the degree of motor neuron damage in ALS, but the abnormal increase of F wave and H wave is rarely found in patients with late ALS. The abnormal degree of F wave and H wave in ALS is not as obvious as that of EMG and MEP, but F wave and H wave can reflect the functional state of upper and lower motor neurons and are the supplement of EMG and MEP.

In the process of clinical detection and diagnosis, EMG examination is an important basis for the diagnosis of ALS. The results of our study showed that the sensitivity of EMG detection was 76.56%, the specificity was 78.33%, and the AUC was 0.8578. It showed that EMG detection of ALS had better diagnostic value. If ALS is highly suspected, EMG is preferred. EMG must select four areas for muscle examination, which should include brain stem (select at least one piece, such as sternocleidomastoid muscle, tongue muscle, facial muscle, or masticatory muscle), neck segment (at least two upper limb muscles), chest segment (T. lower paraspinal muscle or rectus abdominis muscle), and lumbosacral segment (at least two lower limb muscles). If you want to understand the upper motor nerve involvement, choose MEP. If you want to know the degree of upper and lower motor neurons involved, you can choose F wave and H wave; MCV is mainly used for differential diagnosis of ALS. Neuroelectrophysiological technology plays an important role in the diagnosis of ALS, but because of the diversity of clinical manifestations and the complexity of diagnosis and differential diagnosis of ALS, it is necessary to closely combine clinical comprehensive analysis and follow-up.

In conclusion, patients with clinically suspected ALS should undergo electrophysiological testing as soon as possible. Electrophysiological testing is conducive to the early diagnosis and differential diagnosis of ALS.

## Figures and Tables

**Figure 1:** Determination of EMG value.

**Figure 2:** Determination of MEP value.

**Figure 3:** Comparison of results of F wave and H wave in ALS group.

**Figure 4:** Comparison of abnormal rates of nerve conduction values in ALS.

**Figure 5:** ROC curve analysis of electrophysiological detection of ALS.

The article "Study on the Diagnostic Value of Neuroelectrophysiological Examination in Patients with Amyotrophic Lateral Sclerosis" was retracted in 2023. Reasons: signs of a paper mill; compromised peer review; unreliable results or conclusions.

## Data Availability

Data generated in this study are available from the corresponding author under reasonable requests.
